# The Patterns of Non-adherence to Medication in the Management of Cardiovascular Disease: A Descriptive Study

**DOI:** 10.7759/cureus.69810

**Published:** 2024-09-20

**Authors:** Anurag Agarwal, Shilpa Mannagudda Sandip, Amey Joshi, Arshitha Ashok

**Affiliations:** 1 General Surgery, Betsi Cadwaladr University Health Board, Bangor, GBR; 2 Community Medicine, Vydehi Institute of Medical Sciences and Research Centre, Bangalore, IND; 3 Internal Medicine, Sparrow Hospital-Michigan State University, East Lansing, USA; 4 Ophthalmology, Jagadguru Jayadeva Murugarajendra (JJM) Medical College, Davanagere, IND

**Keywords:** adherence, cardiovascular disease, medical therapy, systemic hypertension, treatment regimen

## Abstract

Introduction: Cardiovascular diseases (CVDs) such as hypertension, ischemic heart disease, and stroke are highly prevalent and have a significant impact on quality of life and the healthcare economy. This study aimed to evaluate adherence to medication regimens in CVD patients.

Materials and methods: A cross-sectional descriptive study of 203 patients was conducted using a semi-structured questionnaire which included an eight item Morisky Medication Adherence Scale (MMAS-8) to assess medication compliance.

Results: The survey included 203 patients, 164 (81%) males and 39 (19%) females. Overall, 156 (76.8%) had medical insurance, while only 47 (23.2%) were not medically insured. In total, 161 patients (79.3%) adhered to the medical regimen.

Conclusion: Most participants adhered to their treatment regimen in the present study. However, inadequate knowledge regarding side effects and abrupt discontinuation of medications without physician consultation was reported to a high degree. These findings highlight the areas for improvement in healthcare to improve medication adherence rates.

## Introduction

Cardiovascular diseases (CVD) account for nearly 40.8 million disability-adjusted life years (DALYs) every year. These diseases are a heavy burden on the economies of low- and middle-income countries [1]. Poor medication adherence significantly contributes to increased cardiovascular events [2]. Myocardial infarction, stroke, heart failure, and hypertensive heart disease are common CVDs where medication compliance is crucial to prevent associated adverse cardiac events, hospitalization, and mortality [2,3]. Recent studies have also found that between 33% and 66% of all medication-related hospital admissions are attributed to non-adherence [2]. Most commonly used medications in cardiovascular disease include, but are not limited to, angiotensin-converting enzyme (ACE) inhibitors, angiotensin receptor blockers (ARBs), beta-blockers, calcium channel blockers (CCBs), aspirin, and diuretics. This study was conducted to evaluate the rates of medication non-compliance in cardiovascular disease (including ischemic heart disease {IHD}, hypertension {HTN}, and stroke) in low-income backgrounds to suggest directed strategies to overcome these limitations.

## Materials and methods

A cross-sectional descriptive study was conducted among 203 patients. The inclusion criteria were (1) age of 18 years and above; (2) a diagnosis of hypertension, ischemic heart disease, and stroke; and (3) being on prescribed medical therapy for at least six months. The exclusion criteria were (1) patients who were critically ill, and (2) those unable to provide consent for the study. Hypertension was defined as per the National Institute for Health and Care Excellence (NICE) guidelines as follows: clinic systolic blood pressure sustained at or above 140 mmHg, diastolic blood pressure sustained at or above 90 mmHg, or both; and subsequent ambulatory blood pressure monitoring (ABPM) or home blood pressure monitoring (HBPM) at or above 135/85 mmHg [4]. IHD was defined based on a history of cardiac angiography findings that demonstrated a significant stenosis of the coronary arteries [5]. Stroke was defined as a clinical syndrome of presumed vascular origin characterized by rapidly developing signs of focal or global disturbance of cerebral functions that last longer than 24 hours or lead to death [6].

The data were collected using a pre-designed semi-structured questionnaire (figures in appendix). The questionnaire was presented to the participants after seeking written informed consent and those who met the inclusion criteria. The participants were chosen by convenient sampling technique from those who visited the outpatient clinic in the Department of General Medicine and Department of Cardiology. Data collected included demographic information (age, gender, occupation, socioeconomic status calculated as per modified BG Prasad Scale, and availability of health insurance) and treatment adherence and reason for non-adherence, which was then measured using the eight-point Morisky Medication Adherence Scale (MMAS) [7,8]. The first seven items were yes/no responses, while the last included questions based on medication-taking behaviors. Based on the summated scores from the MMAS-8 ranging from 0 to 8, the scoring criteria of the scale and cut-points are predetermined, and adherence levels were categorized as high (=8 points), medium (6 or 7 points), and low (<6 points). The sensitivity and specificity of the eight item scale are 93% and 53%, respectively [9]. Written informed consent was obtained from all participants. The data were analyzed using SPSS version 23 (Armonk, NY: IBM Corp.). The data were presented as frequencies and percentages, and the association between variables was tested using the chi-square test, and p <0.05 was taken as statistically significant. The study was approved by the Institutional Ethics Committee of Vydehi Institute of Medical Sciences and Research Centre (#VIEC/2017/APP/068).

## Results

The current study included 203 patients. Table 1 lists demographic details. In this study, males were the predominant gender (n=164, 81%), 115 of 203 participants (56.6%) were between the age of 40 and 60 years, and 45 participants (22.2%) were unemployed. In this study, adherence was highest among professional workers (n=52, 92.8%), and the lowest adherence was among unemployed (n=21, 80.7%) (Table 2). The majority of participants, 161 (79.3%), were found to be compliant with their medication regimen, whereas 42 (20.7%) were not compliant with their medication regimen. Of the 42 participants, 38% (n=16) respondents were found to be non-compliant with their medications due to financial constraints, 38% (n=16) due to forgetfulness, due to no perceived improvement in their medical condition, and 4.7% (n=2) due to side effects of their particular medications (Table 3). Eight items Morisky Medication Adherence Scale was performed on all the participants as follows: 154 (75.9%) had a high adherence (score of 8), 17 (8.4%) had moderate adherence (score between 6 and 8), and 32 (15.7%) had low adherence (score less than 6) (Table 4).

**Table 1:** Distribution of the study subjects according to the association between adherence to therapeutic regimen and demographic variables. *Adherence to therapeutic regimen according to the Morisky Medication Adherence Scale. P-value <0.05 was considered statistically significant.

Variables	Low adherence*, n (%)	Moderate adherence*, n (%)	High adherence*, n (%)	Total, n (%)	Chi-square value	p- Value
Age						
18-40 years	1 (12.5)	2 (25)	5 (62.5)	8 (3.9)	8.286	0.102
40-60 years	12 (10.4)	7 (6.1)	96 (83.5)	115 (56.6)		
60-80 years	14 (18.6)	8 (10.6)	53 (70.8)	75 (36.9)		
>80 years	5 (100)	0 (0)	0 (0)	5 (2.6)		
Total	32 (15.7)	17 (8.4)	154 (75.9)	203 (100)		
Gender						
Male	27 (16.4)	13 (7.9)	124 (75.7)	164 (80.8)	0.998	0.210
Female	5 (12.8)	4 (10.2)	30 (77)	39 (19.2)		
Total	32 (15.7)	17 (8.4)	154 (75.9)	203 (100)		
Health insurance						
Yes	5 (3.2)	5 (3.2)	146 (93.6)	156 (76.8)	3.153	0.01
No	27 (57.5)	12 (25.5)	8 (17)	47 (23.2)		
Total	32 (15.7)	17(8.4)	154 (75.9)	203 (100)		

**Table 2:** Distribution of the study subjects according to the association between adherence to therapeutic regimen and sociodemographic variables. *Adherence to therapeutic regimen according to the Morisky Medication Adherence Scale. P-value <0.05 was considered statistically significant.

Variables	Low adherence*, n (%)	Moderate adherence*, n (%)	High adherence*, n (%)	Total, n (%)	Chi-square value	p-Value
Occupation						
Professional	2 (3.5)	2 (3.5)	52 (92.8)	56 (27.6)	11.439	0.267
Semi-professional	0 (0)	2 (6.1)	31 (93.9)	33 (16.2)		
Clerical, shop owner, farmer	1 (4.5)	5 (22.7)	16 (72.8)	22 (10.8)		
Skilled worker	0 (0)	3 (6.7)	42 (93.3)	45 (22.2)		
Semi-skilled worker	0 (0)	1 (7.7)	12 (92.3)	13 (6.4)		
Unskilled worker	8 (100)	0 (0)	0 (0)	8 (3.9)		
Unemployed	21 (80.7)	4 (15.4)	1 (3.9)	26 (12.9)		
Total	32 (15.7)	17 (8.4)	154 (75.9)	203 (100)		
Social class as per modified BG Prasad Socioeconomic Scale 2019 (Rs. per month)						
Class V	16 (14.9)	3 (2.8)	88 (82.3)	107 (52.7)	11.439	0.621
Class IV	0 (0)	4 (28.5)	10 (71.5)	14 (6.9)		
Class III	4 (8.3)	0 (0)	44 (91.7)	48 (23.7)		
Class II	9 (32.1)	10 (35.8)	9 (32.1)	28 (13.8)		
Class I	3 (50)	0 (0)	3 (50)	6 (2.9)		
Total	32 (15.7)	17 (8.4)	154 (75.9)	203 (100)		

**Table 3:** Distribution of the study subjects according to reason for non-adherence to medical therapy. *Adherence to therapeutic regimen according to the Morisky Medication Adherence Scale. P-value <0.05 was considered statistically significant.

Reason for non-adherence	Low adherence*, n (%)	Moderate adherence*, n (%)	High adherence*, n (%)	Total, n (%)	Chi-square value	p- Value
Forgetfulness	12 (75.0)	2 (12.5)	2 (12.5)	16 (38.0)	2.912	0.131
Financial problems	10 (62.5)	5 (31.2)	1 (6.3)	16 (38.0)		
Medicine side effect	1 (50.0)	1 (50.0)	0 (0.0)	2 (4.8)		
Lack of improvement in CVD	3 (75.0)	1 (25.0)	0 (0.0)	4 (9.6)		
Lack of efficacy of medicine	4 (100)	0 (0.0)	0 (0.0)	4 (9.6)		
Total	29 (69.0)	9 (21.4)	4 (9.6)	42 (100)		

**Table 4:** Distribution of the study subjects according to association between adherence and medical regimen prescribed. *Adherence to therapeutic regimen according to the Morisky Medication Adherence Scale. P-value <0.05 was considered statistically significant.

Adherence to doctor’s prescription	Low adherence*, n (%)	Moderate adherence*, n (%)	High adherence*, n (%)	Total, n (%)	Chi-square value	p-Value
Yes	3 (1.9)	8 (4.9)	150 (93.2)	161 (79.3)	45.218	0.04
No	29 (69.0)	9 (21.4)	4 (9.6)	42 (20.7)		
Total	32 (15.7)	17 (8.4)	154 (75.9)	203 (100)		

## Discussion

The present study is a cross-sectional analysis of 203 patients with cardiovascular diseases, which included IHD, HTN, and stroke. The present study reported a high degree of medication compliance with nearly 79% of the study population being adherent to their therapeutic regimen. Non-adherence to CVD medical regimen was commonly seen among the financially lower strata, defined by class V as per the modified BG Prasad Scale for socioeconomic status, comprising 52.7% of the study population. We find this to be a critical finding in our study, as the incidence of CVD has been found to be higher in low-income groups with higher associated mortality [10]. A systemic review done by Chauke et al., which focused mainly on patient groups belonging to low- and middle-income countries showed the main contributory factors to non-adherence were influenced by a lack of knowledge, negative attitudes, and negative beliefs, leading to poor quality of life [11]. Medication non-compliance due to varied reasons may be a contributing factor to the degree of higher CVD incidence and mortality. The availability of insurance was also assessed in the present study as this may be a potential barrier to seeking healthcare and affect medication availability and thereby compliance. In the present study, although the study population mostly involved low-income groups, it was found that the majority of them were medically insured. In Western countries, most of the population avails health insurance, and these trends are rising in India, too [12].

Education on cardiovascular diseases is crucial in its effective management. Hence, health education has to be provided, and awareness should be generated among cardiovascular patients, leading to better disease control and prevention of long-term complications. A systemic review conducted by Kvarnström et al., also concluded that better communication and better information on the disease and its medication is essential to improve adherence to medications [13]. The present study observed that 79.3% of the study population adhered to their medications. The common causes for non-adherence in the present study were forgetfulness and financial constraints, but a small group also reported non-adherence due to side effects of medication and no perceived improvement from medical therapy. Other studies reported high levels of stress, greater complexity of the medical regimen with polypharmacy and poor perceived health status were found to have significantly lower levels of medication adherence [14]. A similar study by Ho et al. suggested that medication non-adherence was associated with higher CVD-related hospitalization and revascularization procedures [15].

Treating chronic illnesses commonly includes the long-term use of pharmacotherapy [16]. After surveying 203 patients, about 42 discontinued their medication without a formal physician consultation. Several studies have confirmed that a low adherence to medical therapy can lead to adverse health outcomes. Thus, in the cardiovascular field, a low adherence has been associated with an increased incidence of target organ damage and cardiovascular events in patients with hypertension [17,18]. Forgetfulness and financial constraints were the leading causes of discontinuation. Abrupt discontinuation of medication may lead to numerous side effects. Patients must be informed of these withdrawal effects, which may lead to improved compliance. Consented reminders, pill counts, prescription refill data, electronic monitoring system, measurement of drug levels, digital medicines, and passive and active communication between the provider and patient were few tips suggested to improve adherence to medications [18,19]. However, further study is required to assess the withdrawal effect of discontinuation of medication.

Limitations

The study had several limitations. This was a single-center descriptive study where the effect of medication adherence to hospitalizations, adverse cardiac outcomes, and mortality could not be measured. Multi-centric prospective studies studying these outcomes will provide further insights into these associations. As the outcomes of this study were obtained through questionnaires, there is a possibility of recall bias and the Hawthorne effect. Lastly, MMSA-8 scale has a high sensitivity rate but a low specificity rate.

## Conclusions

This study observed a high degree of medication compliance in CVD. Forgetfulness due to polypharmacy, financial limitations, and lack of perceived improvement in symptoms with treatment, were reasons for non-compliance. This study highlights potential areas of intervention through regular monitoring of medication compliance in clinic visits, pill-boxes to reduce forgetfulness, counseling regarding secondary preventive strategies, and adverse effects of abrupt discontinuation of therapy. Employing a repetitive teaching strategy may prove advantageous. Moreover, providers should be aware that different socioeconomic strata present distinct challenges to medication adherence. To alleviate the burden on patients, it is essential to strengthen infrastructure, human resources, promote health insurance schemes, and provide affordable generic or alternative medication therapies. Appropriate utilization of mass media, television advertisements and pamphlets for information, education, and communication are crucial.
